This article has been retracted.

# LncRNA LBX2-AS1 promotes colorectal cancer progression and 5-fluorouracil resistance

**DOI:** 10.1186/s12935-021-02209-y

**Published:** 2021-09-17

**Authors:** Yu-Nan Ma, Yong-Gang Hong, Guan-Yu Yu, Si-yuan Jiang, Bo-lun Zhao, An Guo, Yao Wang, Xiao-ming Cui, Li-Qiang Hao, Hao Zheng

**Affiliations:** 1 Key Laboratory of Carcinogenesis and Translational Research (Ministry of Education), Department of Laboratory Animal, Peking University Cancer Hospital & Institute, Beijing, 100142 China; 2 Department of Colorectal Surgery, Changhai Hospital, Second Military Medical University, Shanghai, 200433 China; 3 School of Nursing, Second Military Medical University, Shanghai, 200438 China; 4 School of Nursing, Dalian University, Dalian, 116000 Liaoning China; 5 Department of Reproductive Heredity Center, Changhai Hospital, Second Military Medical University, Shanghai, 200433 China; 6 Shanghai Key Laboratory of Hepatobiliary Tumor Biology (EHBH), Shanghai, 200438 China; 7 State Key Laboratory of Pathogen and Biosecurity, Beijing Institute of Microbiology and Epidemiology, Beijing, People’s Republic of China; 8 Third Department of Hepatic Surgery, Eastern Hepatobiliary Surgery Hospital, Second Military Medical University, Shanghai, 200438 China

**Keywords:** LBX2-AS1, Colorectal cancer, M6A, 5-FU, ceRNA

## Abstract

**Background:**

Recent reports suggest that the long non-coding RNA LBX2 antisense RNA 1 (LBX2-AS1) acts as an important regulator in cancer progression, but its significance in colorectal cancer (CRC) remains undetermined.

**Methods:**

LBX2-AS1 expression levels in CRC were determined from the GEPIA database and CRC tissues to investigate clinical relevance. meRIP-PCR assays investigated the molecular mechanisms underlying the function of m6A in LBX2-AS1. Loss of function experiments was used to define the role of LBX2-AS1 in the progression of CRC. The ceRNA function of LBX2-AS1 was evaluated by RNA immunoprecipitation. In vitro and PDX models were used to determine if LBX2-AS1 promotes 5-fluorouracil resistance.

**Results:**

Data from the TCGA and our institutional patient cohorts established that LBX2-AS1 levels were significantly upregulated in most CRC tissues relative to normal adjacent colon tissues. Moreover, LBX2-AS1 levels were positively correlated with aggressive disease characteristics, constituting an independent prognostic indicator of overall patient survival. Mechanistic investigations suggested that the increased LBX2-AS1 in CRC was mediated by METTL3-dependent m6A methylation. In vitro experiments indicated that knockdown of LBX2-AS1 inhibited CRC proliferation, migration and invasion with this phenotype linked to LBX2-AS1-mediated regulation of AKT1, acting as a ceRNA to sponge miR-422a. Ex vivo analysis of patient-derived CRC xenografts showed that low LBX2-AS1 expression cases exhibited 5-FU responsiveness and clinical investigations confirmed that low LBX2-AS1 expression was associated with improved clinical benefits from 5-FU therapy.

**Conclusions:**

Together these results suggest that LBX2-AS1 may serve as a therapeutic target and predictor of 5-FU benefit in CRC patients.

**Supplementary Information:**

The online version contains supplementary material available at 10.1186/s12935-021-02209-y.

## Background

Colorectal cancer (CRC) is among the most common cancer types worldwide [1], with failure to control disseminated disease typically resulting in patient death [2]. Chemotherapy based on 5-FU alone or in combination with other therapeutic agents is commonly used to treat CRC. However, 5-FU responsiveness is highly variable, and chemoresistance commonly develops in CRC patients, ultimately leading to treatment failure [3, 4]. The mechanistic basis for 5-FU resistance, however, is complex and remains to be fully defined.

Long noncoding RNAs (lncRNAs) are defined as non-protein encoding RNA molecules that exceed 200 nucleotides in length [5–9]. Nonetheless, they principally function as gene regulators, displaying various functional modes including acting as competing endogenous RNAs (ceRNAs) that sponge microRNAs to block their regulatory effects. The levels of lncRNAs are frequently dysregulated in various tumors where they play key roles in initiating or driving tumor development including CRC [10–15].

LBX2 antisense RNA 1 (LBX2-AS1), transcribed from the intron of chromosome 2p13.1, is a newly discovered lncRNA which was initially reported to act as a tumor promoter and predict poor prognosis of esophageal squamous cell carcinoma patients [16]. Moreover, it was reported that upregulation of LBX2-AS1 enhanced the proliferation of gastric cancer via a miR-219a-2-3p/FUS/LBX2 axis [17]. A separate ceRNA function was also revealed where LBX2-AS1 was shown to sponge miRNA-384 to increase IRS1 expression and promoting hepatocellular carcinoma growth [18]. Furthermore, increased LBX2-AS1 levels were associated with poor prognosis in non-small cell lung cancer and shown to promote disease progression via Notch signaling [19]. However, whether LBX2-AS1 fulfils similar roles in CRC progression was not currently known. On this basis, we investigated the impact of LBX2-AS1 in CRC cancer, establishing that LBX2-AS1 expression was associated with poor patient outcomes. We then sought to identify the molecular mechanisms involved and uncovered a novel role for LBX2-AS1 in driving CRC pathogenesis and drug resistance.

## Methods

### Patients and clinical specimens

A total of 256 CRC tissues were utilized from patients undergoing surgery at Changhai hospital between 2008 and 2013 (Cohort A). Complete follow-up information was available and used to evaluate LBX2-AS1 expression and survival analysis. A total of 53 primary CRC patients that received 5-FU therapy after surgery at Changhai hospital from 2013 to 2015 (Cohort B) were employed to evaluate LBX2-AS1 expression and 5-FU sensitivity. A further 192 patients (Cohort C) received 5-FU therapy after surgery at Changhai hospital from 2009 to 2013 with complete follow-up information for survival analysis. Detailed clinicopathological information is provided in Table 1. Ethical approval for this study was provided by The Ethics Committee of Changhai hospital.

**Table 1:** Association between LBX2-AS1 protein expression and clinicopathologic characteristics of 265 CRC patients in the study cohort

Characteristics	No.of	LBX2-AS1 protein level		P value
	Patient	High (N = 135)	Low (N = 130)	
Gender				0.182
Female	117	65	52	
Male	148	70	78	
Age (years)				0.641
< 60	76	37	39	
≥ 60	189	98	91	
Tumor location				0.441
Rectum	118	57	61	
Colon	147	78	69	
Differentiation grade				0.330
Well + moderate	201	99	102	
Poor	64	36	28	
Tumor size (cm)				0.259
< 5	105	49	56	
≥ 5	160	86	74	
Local invasion				**0.014**
pT1–T2	201	95	116	
pT3–T4	64	40	24	
Lymph node metastasis				**0.031**
N0 + N1	164	75	89	
N2	101	60	41	
TNM stage				**0.017**
I + II	158	71	87	
III	107	64	43	
Adjuvant chemotherapy				0.245
No	76	43	33	
Yes	189	92	97	
CA19-9(kU/L)				0.251
< 40	123	58	65	
≥ 40	142	77	65	
Serum CEA level (ng/mL)				0.730
< 10	117	61	56	
≥ 10	148	74	74	

Bold type indicates statistical significance

### qRT-PCR

RNA was extracted from samples using the miRNeasy Mini-kit (#217004, Qiagen, Xuhui, Shanghai, China), after which Reverse Transcriptase (AP101-01, Transgene, Xuhui, Shanghai, China) was used to prepare cDNA. A 7300-sequence detection system (Takara) was used to conduct qRT-PCR reactions with SYBR Green Master Mix (cat. no. RR716; Takara Biotechnology Co., Ltd.) using 35 cycles of 12 s at 95 °C and 1 min at 60 °C. For normalization, GAPDH or U6 was used as endogenous control genes. The primers used are listed in Additional file 1: Table S1.

### Cell culture

Two CRC cell lines (HCT116 and SW480) were obtained from the American Type Culture Collection (Manassas, VA, USA) and grown in Dulbecco’s modified Eagle’s medium (DMEM; Gibco; Thermo Fisher Scientific, Inc., Waltham, MA, USA) supplemented with 10% heat-inactivated fetal bovine serum (FBS; Gibco; Thermo Fisher Scientific, Inc.), 100 U/mL penicillin, and 100 mg/mL streptomycin (Gibco; Thermo Fisher Scientific, Inc.). The cells were maintained at 37 °C in a humidified atmosphere comprising 5% CO_2_.

### Cell transfection

For loss-of-function studies, small interfering RNA (siRNA) specifically targeting METTL3, METTL14, WTAP, FTO, ALKBH5, IGF2BP1/2/3, YTHDF1/2/3 (si-#1,2), LBX2-AS1 (si-#1,2,3) and nontargeting control siRNAs (si-NC) were obtained from Guangzhou RIBOBIO Co., Ltd (Guangzhou, China). Lentiviral expression vectors encoding AKT1 (LV-AKT1) and controls (LV-NC) were obtained from Shanghai GenePharma Co., Ltd (Shanghai, China). Agomirs targeting miR-422a (agomir-422a) and the negative control (agomir-NC) were designed and generated by GenePharma Co., Ltd (Shanghai, China). miR-422a antagomir (antagomir-422a) was used to silence endogenous miR-422a expression, and antagomir-NC was used as the control for antagomir-422a. Cells were seeded into 6-well plates one day before transiently transfecting the aforementioned reagents into cells using Lipofectamine 2000™ (LIFE 11668-019, Invitrogen; Thermo Fisher Scientific). siRNA sequences are detailed in Additional file 1: Table S2.

### Cell proliferation assays

Cell proliferation was measured using the CCK-8 assay as previously described [20]. Cells were seeded into 96 well plates (2 × 10^3^ cells/well) and cultured for 1–4 days before the addition of 3-(4, 5-dimethyl-2-thiazolyl)-2, 5-diphenyl-2-H-tetrazolium bromide (20 μL/well). After 20 min incubation the reactants were dissolved in DMSO (200 μL/well) and OD values at 490 nm measured using an automated plate reader (Bio-Rad Laboratories, CA).

### Transwell invasion assays

Migration and invasion assays, respectively, were performed with uncoated or Matrigel coated Transwell chambers (Corning) as previously described [21]. Briefly, CRC cells (2 × 10^4^ cells) in 200 μL volume were added to the top chamber and the bottom chamber filled with culture medium containing 20% FBS (600 μL). After 18 h, the inserts were stained with crystal violet and the number of invading CRC cells enumeration using an inverted microscope (Carl Zeiss, Germany).

### RNA immunoprecipitation (RIP) assay

The Magna RIP RNA-Binding Protein Immunoprecipitation Kit (#17-701, Millipore, Bedford, MA, USA) was used to perform RIP assays as previously described [21].

### Luciferase reporter assay

The fragments of LBX2-AS1 comprising wild-type (WT) and mutant (MUT) miR-422a binding sites were designed and synthesized by Shanghai GenePharma and luciferase reporter assays performed as previously described [21].

### Experimental animal models

For the PDX model, fresh patient CRC tissues were cut into fragments with a volume of 3 × 3 mm^3^ and then implanted subcutaneously into the flanks of nude mice. The mice were given 5-FU (30 mg/kg) or vehicle orally twice a week for 24 days. Tumor growth was measured at the indicated time points. After 24 days, the mice were sacrificed for euthanasia by intraperitoneal injection of Pelltobarbitalum Natricum (150 mg/kg). All procedures involving animals were approved by the Ethics Committee of Peking University Cancer Hospital & Institute.

### LBX2-AS1 degradation rate

The rate of mRNA degradation of LBX2-AS1 was assessed in the presence of the transcription inhibitor actinomycin D as previously described [22].

### m^6^A meRIP-qPCR

MeRIP assays were performed following the manufacturer’s instructions (Magna MeRIP m6A Kit).

### Statistical analysis

SPSS 17.0 (SPSS Inc, IL, and USA) was used for statistical analysis. The statistical method used is described in the Figure legends with P < 0.05 set as the significance threshold. All experiments were repeated at least three times.

## Results

### LBX2-AS1 expression is elevated in CRC patient tumors and correlates with clinical characteristics

We first analyzed the CRC TCGA dataset using the online tool GEPIA. This analysis revealed that LBX2-AS1 expression was increased in CRC tissues compared to normal tissues (Foldchange > 1.5, P < 0.05, Fig. 1A), and moreover, LBX2-AS1 exhibited gradually increasing expression from Stage I to IV CRC tissues (Fig. 1B). We next sought to independently verify these data in cohort A consisting of 256 paired CRC tissues and adjacent normal tissues. As shown in Fig. 1C, D, the expression of LBX2-AS1 in CRC samples was increased relative to control tissues, with 198/256 (77.3%) of CRC tissues exhibiting significantly higher LBX2-AS1 expression. Based on these data, we divided the 265 patient CRC samples according to their median levels of LBX2-AS1 expression (LBX2-AS1-high or -low; n = 135 and 130, respectively). Univariate analysis against clinicopathological characteristics revealed that higher LBX2-AS1 levels were associated with local invasion of pT3-T4 (P = 0.014), the presence of lymphatic metastasis (P = 0.031), and more advanced TNM stage (P = 0.017) (Table 1). Based on these data we then turned to consider the impact of LBX2-AS1 on patient outcomes.

**Fig. 1:** Expression of lncRNA LBX2-AS1 in CRC. **A** Analysis using the online tool GEPIA indicated that LBX2-AS1 expression was increased in CRC samples relative to normal tissues. **B** Expression of LBX2-AS1 in CRC tissues according to TNM stage using GEPIA. **C**, **D** qRT-PCR was used to assess LBX2-AS1 expression in 265 paired normal and CRC tumor tissues (cohort A). For **A** and **C**, mean ± s.e.m. were derived from n = 3 independent experiments *P < 0.05; ***P < 0.001; Student’s t-test. *COAD* Colon adenocarcinoma, *READ* Rectum adenocarcinoma

### LBX2-AS1 offers prognostic utility in CRC patients

Analysis of CRC data using GEPIA indicated that high LBX2-AS1 levels were associated with poor overall survival (OS) (Fig. 2A); intriguingly however, there were no significant differences indicated for disease-free survival (DFS) (Fig. 2B). Consistently, analysis of data from cohort A also revealed a significant association between elevated LBX2-AS1 expression and reduced OS (Fig. 2C) but not DFS (Fig. 2D). Why LBX2-AS1 expression affects OS but not DFS is unclear but nonetheless, the correlation between higher levels of the lncRNA and worse overall survival suggest LBX2-AS1 has prognostic value. Indeed, a multivariate analysis conducted to identify factors predictive of OS revealed that elevated LBX2-AS1 expression independently predicted reduced OS in CRC patients (Table 2).

**Fig. 2:** CRC patient survival is associated with LBX2-AS1 expression levels. **A** Kaplan–Meier analysis using the online tool GEPIA indicated that patients whose CRC tissues had high LBX2-AS1 expression exhibited significantly reduced overall survival relative to LBX2-AS1-low expressing cases. **B** Analysis of disease-free survival in the dataset from **A** showed no significant differences between high and low LBX2-AS1 expressing cases. **C** Kaplan–Meier analysis of CRC patients from cohort A showing high LBX2-AS1 CRC expression cases exhibited significantly reduced overall survival relative to LBX2-AS1-low expression cases (P = 0.003). **D** Analysis of disease-free survival in the dataset from **C** showed no significant differences between high and low LBX2-AS1 expressing cases. For **A**–**D**, log rank test

**Table 2:** Univariate and multivariate analyses of LBX2-AS1 expression and patients' survival in the study cohort

Variables	Categories	Umivariate analysis				Multivariate analysis			
		HR	95%Cl		P value	HR	95%Cl		P value
Overall survival									
Gender	Male/female	1.236	0.335	2.397	0.808	–	–	–	NA
Age (years)	≥ 60/< 60	0.961	0.763	1.861	0.477	–	–	–	NA
Tumor location	Colon/rectum	1.412	0.297	2.223	0.125	–	–	–	NA
Tumor size (cm)	≥ 5/< 5	1.692	1.396	2.235	0.039	1.247	0.797	1.571	NS
Differentiation grade	Poor/well + moderate	1.593	1.456	4.153	0.013	1.981	1.446	3.332	0.034
Local invasion	pT3–4/pT1–2	1.588	2.122	4.672	0.009	1.531	1.361	1.861	0.038
Lymph node metastasis	N2/N0 + N1	1.954	1.368	2.661	0.034	1.654	1.182	2.151	0.036
TNM stage	III/I + II	2.181	1.632	3.326	0.018	1.992	1.538	3.034	0.016
CA19-9 (KU/L)	≥ 37/< 37	1.041	0.406	1.668	0.152	–	–	–	NA
CEA (ng/mL)	≥ 5/< 5	1.368	0.955	2.174	0.075	–	–	–	NA
LBX2-AS1 level	High/low	3.157	1.823	5.544	0.011	1.675	1.211	2.841	0.022
Disease-free survival									
Gender	Male/female	1.334	0.577	1.941	0.373	–	–	–	NA
Age (years)	≥ 60/< 60	1.231	0.361	1.834	0.286	–	–	–	NA
Tumor location	Colon/rectum	1.279	0.618	1.884	0.823	–	–	–	NA
Tumor size (cm)	≥ 5/< 5	1.515	1.481	3.346	0.031	0.913	0.745	2.003	NS
Differentiation grade	Poor/well + moderate	1.912	1.717	3.038	0.021	1.957	1.307	3.057	0.045
Local invasion	pT3–4/pT1–2	1.564	1.254	2.885	0.015	1.114	0.977	1.932	NS
Lymph node metastasis	N2/N0 + N1	1.805	1.402	3.366	0.038	1.992	1.334	2.382	0.039
TNM stage	III/I + II	2.155	1.623	3.135	0.028	1.161	0.887	2.112	NS
CA19-9 (KU/L)	≥ 37/< 37	1.291	0.752	2.684	0.653	–	–	–	NA
CEA (ng/mL)	≥ 5/< 5	1.317	0.802	2.793	0.438	–	–	–	NA
LBX2–AS1 level	High/low	0.738	0.302	1.543	0.328	–	–	–	NA

*HR* hazard ratio, *95% CI* 95% confidence interval

### m^6^A RNA methylation mediates LBX2-AS1 increased in CRC

To explore the underlying regulatory mechanism whereby LBX2-AS1 was increased in CRC, we treated CRC cell lines with DNA methylation or HDAC inhibitors. As shown in Additional file 1: Figure S1A, these data suggested that LBX2-AS1 expression was not influenced by DNA methylation or histone acetylation. Moreover, RNA interference to downregulate Dicer, the enzyme controlling microRNA processing, also failed to influence the expression of LBX2-AS1 in CRC cells (Additional file 1: Figure S1B). We then turned to consider the involvement of RNA methylation which has emerged as a widespread regulatory mechanism that controls gene expression. Comparing the effects of various so-called m^6^A writers using siRNA-mediated knockdown revealed that inhibition of the METTL3 methyltransferase but not METTL14, or WTAP remarkably decreased the expression of LBX2-AS1. Additionally, knockdown of the m^6^A demethylases FTO or ALKBH5 did not significantly influence the expression of LBX2-AS1 (Fig. 3A and Additional file 1: Figure S1C). Together these data suggest that m^6^A modification by METTL3 was involved in regulating the increased levels of LBX2-AS1 in CRC cells.

**Fig. 3:** m^6^A RNA methylation mediates LBX2-AS1 increased in CRC. **A** qRT-PCR analysis of LBX2-AS1 levels in the indicated CRC cell lines. **B** Identification of the specific m6A methylation loci of LBX2-AS1 using the SRAMP website. **C** m6A levels in LBX2-AS1 were measured by m6A-qPCR in CRC cells transfected with control (sh-NC) or METTL3 targeting (sh-METTL3) shRNAs. **D** qRT-PCR analysis of LBX2-AS1 levels relative to ACTIN in CRC cells treated with actinomycin D (10 μM). **E** qRT-PCR analysis of the level of LBX2-AS1 in the indicated CRC cell lines. **F** RIP assay carried out using anti-IGF2BP1 antibodies. For A, C, D, E and F, mean ± s.e.m. were derived from n = 3 independent experiments *P < 0.05; ^#^P > 0.05; Student’s t-test

To identify the specific m^6^A methylation loci of LBX2-AS1, we interrogated the LBX2-AS1 sequence using the SRAMP website (http://www.cuilab.cn/sramp/), finding 2 positions with a likely abundance of m6A methylation loci (Fig. 3B). Thereafter, m6A-qPCR was then used to confirm the abundance of m6A methylation in these positions and, furthermore that METTL3 induced LBX2-AS1 m6A hyper-methylation in the CRC cell lines (Additional file 1: Figure S1D and Fig. 3C). Our results confirm that silencing of METTL3 reduces mRNA of LBX2-AS1 stability in CRC cells (Fig. 3D).

Our data showed that the interference of IGF2BP1, instead of IGF2BP2, IGF2BP3, YTHDF2, YTHDF3, or YTHDC2 resulted in significant decreases in LBX2-AS1 mRNA in CRC cells (Additional file 1: Figure S1E and Fig. 3E). Furthermore, RNA immunoprecipitation assays suggested the recognition and binding of IGF2BP1 with LBX2-AS1 mRNA in CRC cells (Fig. 3F), proposing that METTL3 induced LBX2-AS1 m6A hypermethylation to enhance its mRNA stability in CRC.

### Knockdown of LBX2-AS1 suppresses CRC cell proliferation and migration

To explore the role of LBX2-AS1 in CRC progression, we first generated shRNAs specific to LBX2-AS1 (sh-LBX2-AS1) to silence the endogenous LBX2-AS1 expression in CRC cells. The high expression of LBX2-AS1 was effectively reduced in HCT116 and SW480 cell lines using sh-LBX2-AS1#2 and these cells were selected for further study (Fig. 4A). Comparative assessment of these cells indicated that LBX2-AS1-knockdown significantly reduced cell proliferation relative to the control cells (Fig. 4B–D). Further analysis using Transwell assays indicated the migratory and invasive capabilities of the LBX2-AS1-knockdown cells were also impaired (Fig. 4E, F). Together these results suggest that LBX2-AS1 can enhance CRC metastasis and progression.

**Fig. 4:** Knockdown LBX2-AS1 suppresses CRC proliferation and migration. **A** Verification LBX2-AS1 knockdown (KD, sh LBX2-AS1) in HCT116 and SW480 lines. **B**–**D** LBX2-AS1 loss‐of‐function and its effects on in vitro proliferation (**B**–**D**), migration (**E**) and invasion (**F**), respectively, were performed using HCT116 and SW480 cells. For **A**, **B**, **D**, **E** and **F**, mean ± s.e.m. were derived from n = 3 independent experiments *P < 0.05; **P < 0.01; ***P < 0.001; Student’s t-test

### LBX2-AS1 drives CRC resistance to 5-FU

To examine the possible relationship between CRC treatment resistance and LBX2-AS1, we treated HCT116 and SW480 cells with 5-FU. Instructively we found that LBX2-AS1 was upregulated by 5-FU in a dose-dependent fashion (Fig. 5A). Moreover, as shown in Fig. 5B, the IC50 for 5-FU was decreased following knockdown of LBX2-AS1 in CRC cells. qPCR analyses further revealed that LBX2-AS1 knockdown also resulted in reductions in the expression of P-gp, MRP1, and BCRP mRNA levels (Fig. 5C). Establishing clinical relevance, analysis of cohort B showed that the expression of LBX2-AS1 in CRC tissues was higher in patients who were resistant to 5-FU (Fig. 5D). Collectively these data indicate that LBX2-AS1 drives CRC cell 5-FU resistance.

**Fig. 5:** LBX2-AS1 bolsters CRC cell resistance to 5-FU. **A** The expression of LBX2-AS1 was measured in 5-FU-treated CRC cells (**B**) LBX2-AS1 silencing was conducted in CRC cells. **B** The viability and 5-FU IC50 values were determined for the indicated CRC cells. **C** qPCR was used to assess P-gp, MRP1, and BCRP expression in the indicated cells. **D** LBX2-AS1 expression in 5-FU-sensitive and -resistant CRC patients from cohort B. For **A**–**D**, mean ± s.e.m. were derived from n = 3 independent experiments *P < 0.05; **P < 0.01; ***P < 0.001; Student’s t-test

### LBX2-AS1 increased AKT1 level by sponging miR-422a

Next, we explored the underlying molecular mechanisms of how LBX2-AS1-mediates enhance CRC progression and 5-FU resistance. Notably, from the GEPIA website we found that LBX2-AS1 expression was positively correlated with AKT1 in CRC tissues (Fig. 6A). To establish the possible link between LBX2-AS1 and AKT1, we investigated the levels of AKT1 after silencing of LBX2-AS1. Indeed, we found the levels of AKT1 mRNA were decreased in LBX2-AS1 knockdown CRC cells (Fig. 6B). Based on these findings we hypothesized that LBX2-AS1 acts as ceRNA for a miRNA that otherwise targets AKT1 expression.

**Fig. 6:** LBX2-AS1 increased AKT1 level by sponging miR-422a in CRC. **A** Pearson correlation analysis using the online tool GEPIA indicated a strong positive correlation between the expression of AKT1 and LBX2-AS1 in CRC samples. **B** AKT1 mRNA was quantitated by RT-qPCR in HCT116 and SW480 cells after transfection with si-LBX2-AS1 or si-NC. **C** Bioinformatics analysis revealed the binding sites of miR-422a within LBX2-AS1. **D** miR-422a expression analysis performed using RT-qPCR. **E** Luciferase reporter assays were performed in indicated CRC cell lines. **F** LBX2-AS1 and miR-422a was enriched in Ago2-immunoprecipitates compared with the IgG control. **G** RT-qPCR detection of miR-422a expression in HCT116 and SW480 cells after transfection with antagomir-422a or antagomir-NC. **H** AKT1 mRNA levels measured by RT-qPCR in the indicated CRC cell lines. **I** P-gp, MRP1, and BCRP mRNA levels measured using RT-qPCR in the indicated CRC cell lines. For **B**, **D**, **E**–**I**, mean ± s.e.m. were derived from n = 3 independent experiments, *P < 0.05; **P < 0.01; ***P < 0.001; ^#^P > 0.05; Student’s t-test

Consistent with this function, subcellular fractionation analysis indicated that LBX2-AS1 was predominantly located in the cytoplasm of CRC cells (Additional file 1: Figure S2). We then focused on exploring the possible regulatory targets of LBX2-AS1 using the open algorithm starBase 3.0 (http://starbase.sysu.edu.cn/). Predictions for miRNAs sharing complementary binding sites in LBX2-AS1 and AKT1 uncovered miR-422a as a likely candidate (Fig. 6C), since miR-422a was previously established to target AKT1 in CRC [23]. To investigate this further, we co-transfected agomiR-NC or agomiR-422a in conjunction with the MUT-LBX2-AS1 or WT-LBX2-AS1 forms into CRC cells for verification in luciferase reporter assays. As expected, transfection with agomiR-422a but not agomiR-NC increased the expression levels of miR-422a in CRC cells (Fig. 6D). Furthermore, agomiR-422a decreased the luciferase activity of the WT-LBX2-AS1 construct in CRC cells but not the activity of the MUT-LBX2-AS1 construct (Fig. 6E). Moreover, RIP assays indicated that LBX2-AS1 and miR-422a were enriched in Ago2-immunoprecipitates relative to the IgG control (Fig. 6F). As shown in Fig. 6G, H, the introduction of antagomiR-422a into LBX2-AS1 knockdown CRC cells was able to reverse the downregulated levels of AKT1 mRNA. Finally, ectopic expression of AKT1 using LV-AKT1 plasmids reversed the downregulation P-gp, MRP1, and BCRP mRNA resulting from knockdown of LBX2-AS1 (Fig. 6I and Additional file 1: Figure S3). Collectively these findings indicate that LBX2-AS1 increases AKT1 levels in CRC by sponging miR-422a.

### LBX2-AS1 expression correlates with patient benefit from 5-FU therapy

Our preceding data suggested separate links between LBX2-AS1 and patient OS and the 5FU resistance of CRC cell lines. To unify these concepts, we finally considered the expression of LBX2-AS1 in cohort C which consists of 87 CRC patients receiving adjuvant 5-FU treatment after surgical resection. Kaplan–Meier analysis revealed that patients with low LBX2-AS1 CRC levels exhibited better OS after 5-FU treatment than patients with high LBX2-AS1 levels (Fig. 7A). We then turned to verify this difference using PDX models derived from patients with differing levels of LBX2-AS1. Notably, PDXs with low LBX2-AS1 levels displayed significant growth inhibition upon 5-FU treatment, while PDXs with high LBX2-AS1 expression did not (Fig. 7B, C). Together these data suggest that LBX2-AS1 expression is correlated with 5-FU response and could be a novel predictor of 5-FU benefit for CRC patients.

**Fig. 7:** Low LBX2-AS1 expression in CRC correlates with patient benefit from 5-FU therapy. **A** Kaplan–Meier analysis showing the overall survival of patients between the high and LBX2-AS1-low expressing groups from cohort C. **B**, **C** PDXs with LBX2-AS1-high and LBX2-AS1-low expression were treated with 5-FU (30 mg/kg body weight) or vehicle for 28 days. Xenografted tumor growth was monitored, and the tumor growth rates were calculated. **D** Working model illustrating how LBX2-AS1-enhances CRC cell malignant phenotypes and promotes 5-FU resistance. For A, log rank test, B and C, *P < 0.05; ^#^P > 0.05, Student’s t-test

## Discussion

Foremost, our study proposes a novel mechanism where the increased levels LBX2-AS1 in CRC cells and patient CRC tissues result from the effects of the METTL3-dependent m^6^A RNA methylation machinery. Increases in LBX2-AS1 expression were correlated with the malignant characteristics of CRC and poor patient survival outcomes. At the primary level, our functional experiments revealed LBX2-AS1 increased the proliferation, migration and invasion of CRC cells. Moreover, LBX2-AS1 acted as ceRNA to sponge miR-422a to increase AKT1 mRNA level to enhance the 5-FU response of CRC cells (Fig. 7D).

Emerging studies have demonstrated that m6A modification of mRNAs plays a critical role in RNA fate, including mRNA stability, splicing, transport, localization, and translation [23, 24]. Methylation of adenosine at the N6 position is mediated by a multicomponent complex composed of METTL3, METTL14, and WTAP in mammals [25, 26]. In contrast, m6A demethylation has been reported to be modulated by FTO and ALKBH5 [27]. Guided by the observation that RNA interference of METTL3 results in decreased LBX2-AS1, our study proposes that LBX2-AS1 expression is regulated by RNA methylation. In addition, we identified that IGF2BP1 was involved in the stabilization of m6A-modified LBX2-AS1 mRNA. To the best of our knowledge, this is the first study to report the involvement of m6A modification in LBX2-AS1 dysregulation in CRC.

The chemotherapeutant, 5-fluorouracil (5-FU), which causes cytotoxic damage, is the basis of standard chemotherapy for CRC and many other cancer types [28]. However, the clinical responses to 5-FU-based chemotherapy, including combined therapy and adjuvant therapy vary greatly, and chemoresistance is a major reason for CRC therapy failure [29, 30]. Therefore, identifying novel biomarkers for patient selection to improve 5-FU efficacy remains a primary unmet need in CRC patient management. Mechanistic studies demonstrated that LBX2-AS1 acted as ceRNA to sponge miR-422a to increase AKT1 expression resulting in the enhanced resistance of CRC cells to 5-FU administration. Consistently, our clinical investigation revealed that patients with low LBX2-AS1 CRC tissue levels were more likely to benefit from 5-FU therapy compared to patients with high LBX2-AS1 levels. This notion was further validated where a correlation was shown between LBX2-AS1 expression and 5-FU responsiveness in PDX models. Here, CRC PDXs with low LBX2-AS1 levels displayed significant growth inhibition upon 5-FU treatment, while PDXs with high LBX2-AS1 levels expression did not respond to 5-FU.

Our study now substantially builds upon previous work showing that LBX2-AS1 is increased in colorectal cancer and promotes proliferation [31]. We reveal that the up-regulation of LBX2-AS1 expression in CRC is related to abnormal levels of m6A modification and moreover, is functionally linked to not only promoting cancer progression but also 5-FU resistance in CRC. With LBX2-AS1 through a ceRNA mode, this was disclosed to occur through a novel miR-422a / AKT1 axis that functions to promote the expression of key drug resistance genes (P-gp, MRP1, BCRP).

## Conclusions

Collectively, these findings suggest that LBX2-AS1 may serve as a predictor of 5-FU benefit in CRC personalized therapy. This promising finding warrants further investigation, both in CRC and in other cancers where LBX2-AS1 is also known to be functionally important.

## Supplementary Information

**Additional file 1: Figure S1.** (A) HCT116 and SW480 cells treated with DMSO, 5-AZA or TSA as indicated were subjected to qPCR analysis of LBX2-AS1 level. (B) HCT116 and SW480 cells transfected with si-Dicer or si-Control as indicated were subjected to r qPCR analysis of LBX2-AS1 level. (C)HCT116 and SW480 cells transfected with the indicated siRNA (si-METTL3, si-METTL14, si-WTAP, si-FTO, si-ALKBH5 or si-Control) were subjected to qPCR assay. (D)The m6A methylation level of Postion-1 and -2 in HCT116 and SW480 cells by m6A-qPCR. (E)HCT116 and SW480 cells transfected with the indicated siRNA (si- IGF2BP-1/-2/-3, si-YTHDF-1/-2/-3 or si-Control) were subjected to qPCR assay. For A-E mean ± s.e.m. were derived from n = 3 independent experiments ∗ P < 0.05; Student’s t-test. **Figure S2.** (A and B) LBX2-AS1 was predominantly located in the cytoplasm of HCT116 (A) and SW480 (B) cells. Mean ± s.e.m. were derived from n = 3 independent experiments. **Figure S3.** HCT116 and SW480 cells transfected with LV-AKT or LV-NC were subjected to qPCR assay. Mean ± s.e.m. were derived from n = 3 independent experiments ∗ P < 0.05; Student’s t-test. **Table S1.** Sequences of primers used in this study. **Table S2.** Target sequences of siRNAs or shRNAs used in this work.

## Data Availability

All data generated or analyzed during this study are included in this published article. The datasets used and/or analysed during the current study are available from the corresponding author on reasonable request.

## Abbreviations

CRC: Colorectal cancer
LBX2-AS1: LBX2 antisense RNA 1
m6A: *N*6-Methyladenosine
